# Diagnostic Value and Prognostic Significance of Procalcitonin Combined with C-Reactive Protein in Patients with Bacterial Bloodstream Infection

**DOI:** 10.1155/2022/6989229

**Published:** 2022-08-11

**Authors:** Yan Zhang, Mei La, Jihong Sun, Mimi Chen, Dandan Liu, Xiaolin Liu, Yating Kang

**Affiliations:** ^1^Clinical Laboratory Northwest A&F University Hospital, Yangling 721000, China; ^2^Yan'an University Xianyang Hospital, Clinical Laboratory, Xianyang, 712000, China

## Abstract

**Objective:**

To study the clinical values and implications for the prognosis of procalcitonin (PCT) combined with C-reactive protein (hs-CRP) in patients with bacterial bloodstream infection.

**Methods:**

One hundred and twenty patients with infection hospitalized from Mar. 2020 to Jun. 2021 were chosen as subjects. All participants were tested for serum PCT, hs-CRP, and blood culture. According to the types of pathogenic bacteria, they were divided into the gram-negative bacteria bloodstream infection group (*n* = 53) and the gram-positive bacteria bloodstream infection group (*n* = 31). Depending on the prognostic outcome of the participants after 28 days, they were categorized into survival and fatality cohorts. The PCT and hs-CRP levels were compared to explore diagnostic value implications for the prognosis of the cases with bacterial bloodstream infection.

**Results:**

Serum PCT and hs-CRP values in the positive cohort were higher than those in the negative cohort. The levels of serum PCT and hs-CRP in pulmonary infection were higher than those in the group with negative cases, and the difference was statistically significant (*P* < 0.05). There were 27 gram-positive participants and 9 gram-negative cases in the positive cohort. The serum PCT value of gram-negative bacterial infection was greater than that of gram-positive bacterial infection. The value of serum PCT in the gram-negative bacterial infection group was higher than that in the gram-positive bacterial infection group, and the difference was statistically significant (*P* < 0.05). The areas under the curve (AUCs) of PCT, combination of hs-CRP and PCT, and hs-CRP were 0.946, 0.783, and 0.991, respectively. The combined examination of PCT and hs-CRP was the largest, PCT was the second, and hs-CRP was the lowest. These results indicated that the accuracy of combined detection of PCT and hs-CRP in the diagnostic bloodstream infection was the highest (0.991), followed by PCT (0.946) and the lowest (0.783). The PCT and hs-CRP levels of the survival cohort were lower than those in the death cohort. AUCs of PCT, hs-CRP and PCT, and hs-CRP were 0.848, 0.826, and 0.934, respectively. The combined examination of PCT and hs-CRP was the largest, followed by PCT and hs-CRP. The accuracy of the combination of PCT and hs-CRP was the highest (0.934), followed by PCT (0.848), and the diagnostic accuracy of hs-CRP was the lowest (0.826).

**Conclusion:**

There were significant differences in the levels of PCT and CRP between the gram-positive bacteria group and the gram-positive bacteria group. PCT and CRP have high diagnostic values in predicting the short-term prognosis of patients. PCT and CRP assist clinical diagnosis and guide treatment and play a positive role in early treatment and prognosis evaluation of patients.

## 1. Introduction

Bloodstream infection is one of the severe infectious diseases in clinic, which seriously threatens the life and health of patients [1]. Bloodstream infection is one of the main factors leading to an increase in morbidity and mortality worldwide [2–5]. In 2002, the number of deaths caused by bloodstream infections in the United States exceeded 30000, and the incidence of bloodstream infections continues to increase [6]. Between 2000 and 2010, the mortality rate of septicemia increased by 17% [7]. Recent reports have suggested that septicemia mortality ranges from 34% to 52% [8]. In 2009, the data from a US study showed that one in 23 hospitalized patients in the United States was affected by bloodstream infection, accounting for 4.2%. In the ranking of hospitalization factors, bloodstream infection ranked sixth.

The incidence of BSI has been increasing year by year. Given the high mortality rate of BSI, the length of stay in hospital is longer and the cost of hospitalization is more expensive, to the extent that patients' lives are seriously threatened. Various invasive diagnostic and testing techniques, like trauma and scald, can disrupt the integrity of the body's barrier function, cause a decrease in immune function, and increase the risk of bloodstream infection. In addition, diverse factors, such as prolonged coma, malnutrition, and advanced age, can also increase the prevalence of bloodstream infections. It therefore becomes important and urgent to identify early, rapidly, and accurately the pathogens causing BSI and then to select the appropriate antibiotic treatment.

With the rapid development of biomedical engineering technology, blood culture technology is widely used in clinic and is regarded as the “gold standard” for the diagnosis of BSI. However, this technique still has some limitations, such as the relatively long cycle of detection of pathogenic microorganisms (usually 24-48 hours), which often leads to the loss of the best opportunity for diagnosis and treatment of BSI patients. Therefore, it is of great clinical significance to find reliable and sensitive biomarkers for early diagnosis of BSI.

At present, the main biomarkers that can be used to diagnose BSI are blood routine test (BRE), procalcitonin (PCT), and C-reactive protein (CRP) [8, 9]. Among them, BRE mainly calculates the changed number of blood cells and related parameters, comprehensively analyzes the morphological distribution of blood cells, and judges the blood condition of the body, so as to screen diseases. PCT is the precursor protein of serum calcitonin, which can hardly be detected under normal conditions. The concentration of PCT increases significantly when patients suffer from pathogenic microbial infections (such as bacterial, fungal, and parasite infections) and sepsis, and when there are some autoimmune reactions and viruses, serum PCT levels do not suddenly increase rapidly. When a local bacterial infection, fungal infection, viral infection, or other chronic inflammation occurs in a certain part of the body, it will not cause an increase in the level of PCT [10–12]. CRP is a nonspecific inflammatory protein synthesized through the liver, and its expression is significantly increased when patients are invaded by bacteria or tissue damage. Previous studies have focused on exploring the expression of PCT and CRP between gram-negative bacteria and gram-positive bacteria, but there are few reports on the diagnosis and prognosis of bloodstream infections by PCT and CRP. Therefore, this study analyzed the clinical data of 120 patients to study the diagnostic value of procalcitonin (PCT) combined with high-sensitivity C-reactive protein (hs-CRP) in the diagnosis of bacterial bloodstream infection and its prognostic significance.

## 2. Materials and Methods

### 2.1. General Information

One hundred and twenty patients with infection hospitalized from March 2020 to June 2021 were selected as the objects of study. All patients were tested for serum PCT and hs-CRP and blood culture. Among the 120 patients with infection, there were 62 males and 58 females with ages from 19 to 85 years (mean 45.83 ± 4.23). Our clinic's Professional Conduct Association gave their approval towards this experiment. Every participant provided written informed consent.

#### 2.1.1. Selection Criterion

(1) There was no limitation to the sex of the patient, and the initial disease was caused by pulmonary infection, urinary tract infection, suppurative meningitis, bacillary dysentery, and other infections. Blood culture samples and serum samples were sent for examination at the same time; (2) without cognitive, language, and intellectual impairment and with basic reading and writing ability; (3) the diagnostic criteria of bloodstream infection met the following requirements: fever, chills, and other symptoms; hematological tests find antigenic substances of pathogens; and/or when pathogenic bacteria or fungi were isolated by blood culture, any of the following requirements can be met: (a) the strains of pathogenic bacteria isolated from many times of blood culture are the same, and the results of the drug sensitivity test are the same; (b) the strains of pathogenic bacteria isolated from other infected sites are the same as those of blood culture, and the results of drug sensitivity test are the same; and (c) it was effective to use sensitive antimicrobial agents for the isolated pathogenic bacteria. (4) The clinical data are complete, (5) there was no history of surgery or trauma within 3 months, and (6) there were no autoimmune diseases and hematological diseases.

#### 2.1.2. Exclusion Criteria

The exclusion criteria are (1) patients with severe heart, liver, and renal insufficiency and malignant tumors, (2) patients who had been treated with corticosteroids for a long time, (3) patients with hematological diseases, (4) patients who had a history of taking antibiotics and hormones within 3 months before entering the group, and (5) patients with a history of organ transplantation and immunosuppressant use.

### 2.2. Methods

The levels of serum PCT and hs-CRP were detected in all patients, and blood culture was performed. The sensitivity, specificity, and diagnostic accuracy of three kinds of detection of bloodstream infection were compared to determine their value in early clinical diagnosis and prognosis evaluation of bloodstream infection. The PCT determination kit (electrochemiluminescence) is from Roche Diagnostic products (Shanghai) Co., Ltd., using the Roche automatic electrochemiluminescence immunoassay system. The hs-CRP determination kit (scatter turbidimetry) comes from Shenzhen Pumen Technology Co., Ltd., using the PA-990P specific protein analyzer. The blood culture instrument comes from BacT/ALERT3D automatic Mycobacterium culture and identification system (Merieux). For the identification and drug sensitivity of gram-positive bacteria, VITEKGP was used, with drug sensitivity VITEKAST-GP67. For the identification and drug sensitivity of gram-negative bacteria, VITEKGN was used, with drug sensitivity VITEKAST-GN09.

#### 2.2.1. Observation Index

On the day of admission and 28 days after the patient's admission, the cubital venous blood was drawn in the early morning on an empty stomach and centrifuged at 3000 r/min for 15 min. The upper serum was separated for testing. The PCT value was detected by the chemiluminescence method, and the kit was purchased from Zhengzhou Antu Bioengineering Co., Ltd. The hs-CRP level was detected by immunoturbidimetry, and the kit was purchased from Shenzhen Pumen Technology Co., Ltd. Analyzer Roche 411.

### 2.3. Statistical Analysis

The SPSS22.0 statistical program was used for data analysis. The chi-squared test (*χ*^2^ test) was applied to compare the counting data. The measured data were expressed by *x* ± *s*, the *t*-test was used, and analysis of variance was used to compare multiple-group data. The difference was statistically significant, and the difference was statistically significant (*P* < 0.05). The area under the receiver operating characteristic (ROC) curve was used to evaluate the clinical diagnostic value of PCT, hs-CRP, and combined detection in bloodstream infection and prognosis of patients.

## 3. Results

### 3.1. Comparison of PCT and hs-CRP Levels between the Two Groups

The values of serum PCT and hs-CRP in the group with positive blood culture were higher than those in the group with negative blood culture, and the difference was statistically significant (*P* < 0.05). See Table 1.

### 3.2. The Serum PCT and hs-CRP Values between the Two Groups of Pulmonary Infection by Blood Culture

In the positive blood culture group, the serum PCT value and hs-CRP value of the patients with pulmonary infection were larger than those in the negative blood culture group, and the difference was statistically significant (*P* < 0.05). See Table 2.

### 3.3. The Serum PCT and hs-CRP Values in Patients with Bloodstream Infection Caused by Gram-Positive Bacteria and Gram-Negative Bacteria

In the blood culture positive group, there were 27 cases of gram-positive bacterial infection and 9 cases of gram-negative bacterial infection. The value of serum PCT in the gram-negative bacterial infection group was higher than that in the gram-positive bacterial infection group (*P* < 0.05). See Table 3.

### 3.4. The Bacteria Species and Serum PCT and hs-CRP Values between Gram-Positive Bacteria and Gram-Negative Bacteria

Among the infections of gram-positive bacteria, there were 14 cases of Staphylococcus epidermidis infection, 9 cases of Staphylococcus aureus infection, 2 cases of Streptococcus infection, and 2 cases of Enterococcus infection. Among the patients infected with gram-negative bacteria, there were 4 cases of Klebsiella pneumoniae infection, 3 cases of Acinetobacter baumannii infection, and 2 cases of Escherichia coli infection, and the serum PCT value of gram-negative bacterial infection was greater than that of gram-negative bacterial infection, and the difference was statistically significant (*P* < 0.05). There was no significant difference in serum hs-CRP between gram-negative bacteria and gram-positive bacteria (*P* > 0.05). There was no statistical significance in the comparison of serum PCT and hs-CRP values in patients infected with gram-negative bacteria (*P* > 0.05). There was no statistical significance in the comparison of serum PCT and hs-CRP values in patients infected with gram-positive bacteria (*P* > 0.05). See Table 4.

### 3.5. Diagnostic Value of PCT, hs-CRP, and Their Combination in Bloodstream Infection

The AUCs of PCT, hs-CRP and PCT, and hs-CRP were 0.946, 0.783, and 0.991, respectively (all *P* < 0.05). The area under the joint detection curve of PCT and hs-CRP was the largest, PCT was the second, and hs-CRP was the lowest. The accuracy of combined detection of PCT and hs-CRP in the diagnosis of bloodstream infection was the highest (0.991), followed by PCT (0.946), and hs-CRP was the lowest (0.783). See Table 5 and Figure 1.

### 3.6. The Serum PCT and hs-CRP Levels between Survival Group and Death Group

Of the 36 patients with bacterial bloodstream infection, 29 survived and 7 died. The serum PCT and hs-CRP values in the survival group were lower than those in the death group, and the difference was statistically significant (*P* < 0.05). See Table 6.

### 3.7. The Value of PCT and hs-CRP in Diagnosing the Prognosis and Survival of Patients

ROC curve analysis showed that the AUCs of PCT, hs-CRP and PCT, and hs-CRP were 0.848, 0.826, and 0.934, respectively (all *P* < 0.05). The AUC of combined detection of PCT and hs-CRP was the largest, followed by PCT, and the lowest was hs-CRP. The accuracy of combined detection of PCT and hs-CRP was the highest (up to 0.934), followed by PCT (0.848), and the diagnostic accuracy of hs-CRP was the lowest (0.826). See Table 7 and Figure 2.

## 4. Discussion

Bloodstream infection (BSI) is a general term for septicemia and bacteremia. Septicemia is when bacteria enter the bloodstream and grow, producing large amounts of toxins and metabolites, causing systemic severe infection syndrome. Bacteremia is toxemia in which bacteria enter the bloodstream temporarily but do not cause obvious symptoms of systemic infection. Under certain conditions, bacteremia and septicemia can be converted into each other [13]. The disease lacks characteristic clinical manifestations in the early stage, so it is difficult to be detected. Because of the high specificity of blood culture, it is often used as the first choice for the diagnosis of bloodstream infection. However, blood culture has the following disadvantages: (1) the blood should be collected before medication, and the blood is easy to be contaminated, (2) the positive rate is easily affected by the number of bacteria, and (3) the culture takes a long time, resulting in the lag of the results. Previous studies have shown that C-reactive protein and procalcitonin play an important role in the occurrence and development of bloodstream infection [14, 15].

Recently, a large number of broad-spectrum antibiotics, hormone drugs, and immunosuppressants have been widely used in clinic with the continuous development of invasive diagnosis and treatment technology. C-reactive protein is an acute phase reactive protein, which is mainly released from the liver under the stimulation of interleukin-6 and other cytokines [16]. When the body is infected, CRP can play both anti-inflammatory and proinflammatory effects, mainly because it can mediate the elimination of pathogens and inhibit the interaction between endothelial cells and white blood cells. Therefore, CRP is often used for the early diagnosis of infectious diseases. Studies have shown that CRP can improve the early diagnosis rate of pneumonia [17, 18]. For patients after surgery, CRP can help distinguish acute appendicitis from other noninfectious abdominal pain and predict infection complications after colorectal surgery [19, 20]. However, some studies have shown that the diagnostic value of CRP alone in sepsis is only moderate, and the predicting positive blood culture and disease prognosis are lower than that of procalcitonin and sTREM-1 [21]. In general, CRP levels decrease within 48 hours after anti-infective treatment [22]. Baruah et al. investigated 891 patients with community-acquired septicemia, showing that CRP levels of most patients decreased within 48 hours and serum CRP levels of all patients decreased within 5 days after anti-infection treatment [23].

Procalcitonin, a propeptide of calcitonin, has no hormonal activity and is usually produced by thyroid C cells. In healthy people, almost all calcitonin is converted to calcitonin, so its content in serum is generally lower than that of 0.05 ng/ml. When infection occurs, the content of serum procalcitonin changes at any time [24]. When the symptoms of sepsis are severe, the content of procalcitonin released into the blood is high. When the symptoms of sepsis are mild, the amount of procalcitonin released into the blood is relatively low. Assicot and his colleagues first proposed PCT as a potential biomarker of sepsis and infection in 1993. Some scholars have shown that the advantage of PCT as a biomarker to predict infection lies in its high stability in vitro, and the serum level can increase within 2-3 hours after infection [25]. The study of Wallihan et al. showed that the areas under the ROC curve of PCT predicting sepsis positive blood culture and negative blood culture were 0.96 and 0.89, respectively [26], indicating that PCT can early predict, so as to take effective diagnosis, treatment, and nursing measures in time. Although PCT is closely related to infection, its specificity for infection is not complete [27]. There is evidence that when patients suffer from trauma or other diseases, the value of PCT can also slightly increase [28]. Therefore, it is impractical to use PCT concentration alone to diagnose sepsis. Generally speaking, when the serum PCT content is higher than 2.0 ng/ml, the risk of sepsis or septic shock increases significantly. When the PCT content is between 0.5 and 2.0 ng/ml, the risk rate is at a medium level. When the PCT content is less than 0.5 ng/ml, the risk rate of sepsis is very low. According to the results of a meta-analysis conducted by Jiaqiong et al., the sensitivity and specificity of PCT in the diagnosis of sepsis are 77% and 79%, respectively, and the diagnostic value is poor [29]. Therefore, when using PCT to predict sepsis or diagnose sepsis, it is necessary to make a comprehensive judgment combined with the clinical characteristics of patients and other experimental indicators. CRP is often used in the early diagnosis of infectious diseases [30, 31]. Therefore, this paper studies the diagnostic value of procalcitonin (PCT) combined with C-reactive protein (hs-CRP) in the diagnosis of bacterial bloodstream infection and its significance for the prognosis of patients. There are some limitations to this study. First, the sample size of this study is not large, and it is a single-center study, so bias is inevitable. In future research, we will carry out multicenter, large-sample prospective studies, or more valuable conclusions can be drawn.

In conclusion, there were significant differences in the levels of PCT and CRP between gram-positive bacteria and gram-negative bacteria. PCT and CRP have high diagnostic value in predicting the short-term prognosis of patients. PCT and CRP assist clinical diagnosis and guide treatment and play a positive role in early treatment and prognosis evaluation of patients.

## Figures and Tables

**Figure 1:** ROC curve of PCT and hs-CRP in the diagnosis of bloodstream infection. Note: the AUCs of PCT, hs-CRP and PCT, and hs-CRP were 0.946, 0.783, and 0.991, respectively (all *P* < 0.05). The area under the joint detection curve of PCT and hs-CRP was the largest, PCT was the second, and hs-CRP was the lowest.

**Figure 2:** ROC curve of prognosis and survival of patients diagnosed by PCT and hs-CR. Note: the AUCs of PCT, hs-CRP and PCT, and hs-CRP were 0.848, 0.826, and 0.934, respectively (all *P* < 0.05). The AUC of combined detection of PCT and hs-CRP was the largest, followed by PCT, and the lowest was hs-CRP.

**Table 1:** Comparison of PCT and hs-CRP levels between the two groups.

Grouping	*N*	PCT (ng/ml)	hs-CRP (mg/l)
Blood culture negative group	84	0.48 ± 0.43	24.72 ± 5.36
Blood culture positive group	36	4.93 ± 0.87	35.38 ± 10.54
*t*		37.516	7.340
*P*		<0.05	<0.05

**Table 2:** Comparison of the serum PCT and hs-CRP values between the two groups ($\bar{x}\pm s$).

Grouping	*N*	PCT (ng/ml)	hs-CRP (mg/l)
Pulmonary infection in patients with negative blood culture	53	0.53 ± 0.47	24.56 ± 5.55
Pulmonary infection in patients with positive blood culture	31	5.09 ± 0.93	35.48 ± 10.66
*t*		29.848	6.178
*P*		<0.05	<0.05

**Table 3:** The serum PCT and hs-CRP values in patients with bloodstream infection caused by gram-positive bacteria and gram-negative bacteria ($\bar{x}\pm s$).

Grouping	*N*	PCT (ng/ml)	hs-CRP (mg/l)
Gram-positive bacteria	27	1.67 ± 0.46	37.29 ± 9.48
Gram-negative bacteria	9	6.54 ± 1.26	34.98 ± 11.67
*t*		17.292	0.598
*P*		<0.05	>0.05

**Table 4:** The bacterial species and serum PCT and hs-CRP values between gram-positive bacteria and gram-negative bacteria ($\bar{x}\pm s$).

Grouping	*N*	PCT (ng/ml)	hs-CRP (mg/l)
Gram-positive bacteria	27		
Staphylococcus epidermidis	14	1.61 ± 0.42	37.51 ± 9.23
Staphylococcus aureus	9	1.68 ± 0.44	37.83 ± 9.45
Streptococci	2	1.68 ± 0.03	39.45 ± 4.12
Enterococci	2	1.65 ± 0.02	36.69 ± 3.87
Gram-negative bacteria	*9*		
Klebsiella pneumoniae	*4*	6.35 ± 1.62	34.28 ± 11.95
Acinetobacter baumannii	*3*	6.15 ± 1.72	35.05 ± 11.59
Pseudomonas aeruginosa	*2*	6.61 ± 1.03	34.88 ± 3.41

**Table 5:** Diagnostic efficacy of PCT, hs-CRP, and combined blood culture in patients with bloodstream infection.

Index	AUC (95% CI)	Truncation value	Sensitivity (%)	Specificity degree (%)	Youden index
PCT (ng/ml)	0.946 (0.911~0.974)	1.283	88.61	94.02	0.818
hs-CRP (mg/l)	0.783 (0.681~0.892)	31.684	63.75	92.54	0.557
PCT+hs-CRP	0.991 (0.972~1.000)	304.39	94.18	98.73	0.921

**Table 6:** The serum PCT and hs-CRP levels between the survival group and the death group.

Grouping	*N*	PCT (ng/ml)	hs-CRP (mg/l)
Survival group	29	1.63 ± 0.76	73.28 ± 30.11
Death group	7	4.18 ± 2.04	117.54 ± 44.83
*t*		5.505	3.167
*P*		<0.05	<0.05

**Table 7:** The value of PCT and hs-CRP in the diagnosis of prognosis and survival of patients.

Index	AUC (95% CI)	Truncation value	Sensitivity (%)	Specificity degree (%)	Youden index
PCT (ng/ml)	0.848 (0.733~0.963)	2.406	91.83	80.65	0.736
hs-CRP (mg/l)	0.826 (0.708~0.944)	74.833	88.94	53.57	0.429
PCT+hs-CRP	0.934 (0.854~1.000)	81.421	88.92	94.27	0.647

## Data Availability

No data were used to support this study.

## References

[1] Kern W. V., Rieg S. (2020). Burden of bacterial bloodstream infection—a brief update on epidemiology and significance of multidrug-resistant pathogens. *Clinical Microbiology and Infection*.

[2] Diekema D. J., Hsueh P. R., Mendes R. E. (2019). The microbiology of bloodstream infection: 20-year trends from the SENTRY antimicrobial surveillance program. *Antimicrobial Agents and Chemotherapy*.

[3] Patel P. K., Gupta A., Vaughn V. M., Mann J. D., Ameling J. M., Meddings J. (2018). Review of strategies to reduce central line-associated bloodstream infection (CLABSI) and catheter-associated urinary tract infection (CAUTI) in adult ICUs. *Journal of Hospital Medicine*.

[4] Fowler V. G., Das A. F., Lipka-Diamond J. (2020). Exebacase for patients with Staphylococcus aureus bloodstream infection and endocarditis. *The Journal of Clinical Investigation*.

[5] Falcone M., Bassetti M., Tiseo G. (2020). Time to appropriate antibiotic therapy is a predictor of outcome in patients with bloodstream infection caused by KPC-producing Klebsiella pneumoniae. *Critical Care*.

[6] Li Y. L., Zhai L. C., Ji J. H., Liu L. Y. (2017). Detection of combined procalcitonin and c-reactive protein applied in the diagnosis of bacterial infections. *Journal of Biological Regulators and Homeostatic Agents*.

[7] Aloush S. M., Alsaraireh F. A. (2018). Nurses’ compliance with central line associated blood stream infection prevention guidelines. *Saudi Medical Journal*.

[8] Leng Y., Chen C., Zhang Y., Luo C., Liu B. (2019). Ability of serum procalcitonin to distinguish focus of infection and pathogen types in patients with bloodstream infection. *Annals of Translational Medicine*.

[9] Kargaltseva N. M., Kotcherovets V. I., Mironov A. Y., Borisova O. Y., Burbello A. T. (2019). Inflammation markers and bloodstream infection (review of literature). *Klinicheskaia Laboratornaia Diagnostika*.

[10] Liang P., Yu F. (2022). Value of CRP, PCT, and NLR in prediction of severity and prognosis of patients with bloodstream infections and sepsis. *Frontiers in Surgery*.

[11] Xiaolei S., Rui Z., Kaiyu F. (2021). The value of IL-17, PCT/ALB and mHLA-DR in evaluating the condition and prognosis of elderly patients with multi-drug resistant Acinetobacter baumannii infection. *People's Liberation Army Medical Journal*.

[12] Hahn W. H., Song J. H., Kim H., Park S. (2018). Is procalcitonin to C-reactive protein ratio useful for the detection of late onset neonatal sepsis?. *The Journal of Maternal-Fetal & Neonatal Medicine*.

[13] Liu H. H., Zhang M. W., Guo J. B., Li J., Su L. (2020). Procalcitonin and C-reactive protein in early diagnosis of sepsis caused by either Gram-negative or Gram-positive bacteria. *Irish Journal of Medical Science (1971-)*.

[14] Gutiérrez-Gutiérrez B., Morales I., Pérez-Galera S. (2019). Predictive value of the kinetics of procalcitonin and C-reactive protein for early clinical stability in patients with bloodstream infections due to gram negative bacteria. *Diagnostic Microbiology and Infectious Disease*.

[15] Bassetti M., Russo A., Righi E. (2019). Role of procalcitonin in bacteremic patients and its potential use in predicting infection etiology. *Expert Review of Anti-Infective Therapy*.

[16] Bamba Y., Moro H., Aoki N. (2018). Increased presepsin levels are associated with the severity of fungal bloodstream infections. *PLoS One*.

[17] Lin M. F., Sun B., Liu Z. Y., Tang P., Zhang L. J., Wang Y. Y. (2020). Evaluation of the clinical diagnostic value of traditional inflammatory markers and novel biomarkers in intracellular bacterial bloodstream infections. *Cytokine*.

[18] Shukun Q., Jianhua L., Rui L. (2022). The value of serum PCT, CRP and NLR in evaluating the bacterial types of patients with bloodstream infection and its effect on prognosis. *Labelled Immunoassay and Clinical Application*.

[19] Dengju H., Saiping X. (2021). Significance of serum IAP and CRP levels in patients with acute appendicitis. *Continuing Medical Education in China*.

[20] Lin C. T., Lu J. J., Chen Y. C., Kok V. C., Horng J. T. (2017). Diagnostic value of serum procalcitonin, lactate, and high-sensitivity C-reactive protein for predicting bacteremia in adult patients in the emergency department. *PeerJ*.

[21] Shan R. F., Zhu Y. A., Qin J., Chen J. P. (2021). Traditional Chinese medicine for septic patients undergoing ulinastatin therapy. *Medicine*.

[22] Jones J. F., Le J., Lee K. C. (2021). Effect of antidepressant use on length of hospitalization in patients on anti-infective therapy. *Journal of Psychiatric Research*.

[23] Baruah A., Paul N. (2021). Abnormal platelet count as a prognostic indicator in community-acquired pneumonia in children. *Indian Journal of Child Health*.

[24] Obaid F. H., Ahmed M. M., Ali M. S., Jasim A. A. (2020). The role of procalcitonin and neutrophilCD64 in non culture-based diagnosis of neonatal and infantile septicemia. *International Journal*.

[25] Ojuawo O. B., Fawibe A. E., Desalu O. O. (2021). Clinical utility of serum procalcitonin in adult patients admitted with community-acquired pneumonia in Ilorin, Nigeria. *Journal of the Pan African Thoracic Society*.

[26] Wallihan R. G., Suárez N. M., Cohen D. M. (2018). Molecular distance to health transcriptional score and disease severity in children hospitalized with community-acquired pneumonia. *Frontiers in Cellular and Infection Microbiology*.

[27] Méndez R., Menéndez R., Cillóniz C. (2018). Initial inflammatory profile in community-acquired pneumonia depends on time since onset of symptoms. *American Journal of Respiratory and Critical Care Medicine*.

[28] Nishikawa H., Shirano M., Kasamatsu Y. (2017). Comparison between procalcitonin and C-reactive protein in predicting bacteremias and confounding factors: a case-control study. *Clinical Chemistry and Laboratory Medicine (CCLM)*.

[29] Ljungström L., Pernestig A. K., Jacobsson G., Andersson R., Usener B., Tilevik D. (2017). Diagnostic accuracy of procalcitonin, neutrophil-lymphocyte count ratio, C-reactive protein, and lactate in patients with suspected bacterial sepsis. *PloS one*.

[30] Ying L., Lin R., Hongfei C. (2022). Application of combined test of whole blood C-reactive protein and blood routine in the diagnosis of bacterial infectious diseases. *Quality Safety and Inspection*.

[31] Ting Y. (2021). Expression and clinical significance of serum PCT, CRP and WBC in patients with severe bacterial infectious diseases. *Chinese Medical Engineering*.

